This article has been retracted.

# PSB0788 ameliorates maternal inflammation‐induced periventricular leukomalacia-like injury

**DOI:** 10.1080/21655979.2022.2061296

**Published:** 2022-04-18

**Authors:** Yilu Li, Dan Wang, Zhuoyang Li, Zhi Ouyang

**Affiliations:** a School of Chemistry and Chemical Engineering, South China University of Technology, scDFG Guangzhou, Guangdong, China; b Department of clinical medicine, Bengbu Medical College, Bengbu, Anhui, China; c Department of clinical medicine, Ningxia Medical University, Yinchuan, Ningxia, China; d South China University of Technology-Zhuhai Institute of Modern Industrial Innovation, Zhuhai, Guangdong, China; e South China University of Technology Hospital, South China University of Technology, Guangzhou, Guangdong, China

**Keywords:** Inflammation, periventricular white matter injury, myelin sheath, PSB0788

## Abstract

Studies have shown that periventricular leukomalacia (PVL) is a distinctive form of cerebral white matter injury that pertains to myelination disturbances. Maternal inflammation is a main cause of white matter injury. Intrauterine inflammation cellular will be propagated to the developing brain by the entire maternal–placental–fetal axis, and triggers neural immune injury. As a low-affinity receptor, adenosine A_2B_ receptor (A_2B_AR) requires high concentrations of adenosine to be significantly activated in pathological conditions. We hypothesized that in the maternal inflammation‐induced PVL model, a selective A_2B_AR antagonist PSB0788 had the potential to prevent the injury. In this work, a total of 18 SD pregnant rats were divided into three groups, and treated with intraperitoneal injection of phosphate buffered saline (PBS), lipopolysaccharide (LPS), or LPS+PSB0788. Placental infection was determined by H&E staining and the inflammatory condition was determined by ELISA. Change of MBP, NG2 and CC-1 in the brain of the rats’ offspring were detected by western blot and immunohistochemistry. Furthermore, LPS-induced maternal inflammation reduced the expression of MBP, which related to the decrease in the numbers of OPCs and mature oligodendrocytes in neonate rats. After treatment with PSB0788, the levels of MBP proteins increased in the rats’ offspring, improved the remyelination. In conclusion, our study shows that the selective A_2B_AR antagonist PSB0788 plays an important role in promoting the normal development of OPCs *in vivo* by the maternal inflammation‐induced PVL model. Future studies will focus on the mechanism of PSB0788 in this model.

## 1. Introduction

Periventricular leukomalacia (PVL) characterized by diffuse demyelination in the white matter of periventricular region [1], is the most common form of white matter injury caused by maternal infection between 23 and 32 weeks of gestation, resulting in impairments in learning, memory, and cognition [2,3]. The mortality associated with PVL is high, with more than 50% of the surviving children developing cerebral palsy [4], including anxiety, inhibitory control and deficits of attention [5–7]. Lately, as perinatal care has improved with modern medical advances in Neonatal Intensive Care Units, the endurance pace of preterm infants at earlier gestational ages has increased [8]. Maternal inflammation is a main cause of white matter injury. Perinatal myelin‐forming oligodendrocytes aggravation prompts a shortfall in white matter development, leading to demyelination‐associated disorders [9].Oligodendrocytes originate from oligodendrocyte precursor cells (OPCs). OPCs differentiate into oligodendrocytes wrap around and myelinate axons, supporting neural signal saltatory conduction across them. Myelin basic protein (MBP) is a primary structural component of myelin and is exclusively expressed in myelin in brain.An intraperitoneal injection of lipopolysaccharide (LPS) into pregnant animals mimics the maternal inflammation caused by a rise in the proinflammatory cytokines level such as interleukin‐1 β (IL‐1 β), interleukin‐6 (IL‐6) and tumor necrosis factor‐α (TNF‐α) [10]. These cytokines propagate the expression of chemokines recruiting neutrophils, monocytes, and macrophages from the maternal circulation to promote intrauterine inflammation [11–13]. Collectively, maternal inflammation is a main cause of white matter injury. Intrauterine inflammation cellular will be propagated to the developing brain by the entire maternal–placental–fetal axis, and triggers neural immune injury [14]. Changes in the subsequent perinatal events cause injury to the developing immune system.The central nervous system development is impacted by the abnormal developing immune system [15]. In this experiment, systemic LPS administration was used to model PVL in pregnant rats. Interestingly, the ultimate common denominator of hypoxia–ischemia and infection is systemic inflammation, leading to brain injury in infants [16–18]. Adenosine A_2B_ receptors (A_2B_AR) are G-protein-coupled receptors, showing relatively lower affinity for adenosine compared to A_1_AR, A_2A_AR, and A_3A_R [19], and also less studied [20]. However, in recent years, significant changes in the level of A_2B_AR have been observed in pathological conditions, such as hypoxia and inflammation [21], where high concentrations of adenosine are required for this receptor to be significantly activated [22]. A_2B_AR is widely distributed in neurons and glial cells of the central nervous system [23]. Recently, Coppi et al found that culturing OPCs with a selective A_2B_AR agonist could lead to decreased expression of proteins associated with the myelin sheath [24], and researchers found that the inhibited A_2B_AR could induce anti-inflammatory responses [25]. In our previous experiments, we found that LPS could significantly increase the expression of A_2B_AR and inhibit the differentiation of OPCs in vitro. PSB0788 is a selective A_2B_AR antagonist that can inhibit A_2B_AR due to its high affinity [26,27]. Therefore, we studied the effects of PSB0788 on the cerebral myelin sheath and oligodendrocytes, at various stages in the newborn rats with inflammation-induced PVL. In this study, it was hypothesized that PSB0788 ameliorates white matter injury via promoting the expression of IL‐10.The aim of the study was to discover new targets for the treatment of PVL. The goal of this study was to prove that PSB0788 could improve the myelination disturbances caused by maternal inflammation‐induced PVL.

## 2. Methods

### 2.1 Animals

Pregnant Sprague-Dawley (SD) rats were provided by the experimental animal center of South China University of Technology(SCUT) and the Laboratory Animal Center of Ningxia Medical University(NMU). Animals were maintained at constant temperature (22 ± 2°C) and humidity (40–60%) at a 12 h:12 h light/dark cycle with free access to food and water. There was one pregnant rat in each cage and all procedures were approved by the Animal Care and Use Committee of NMU.

### 2.2 Grouping

Eighteen pregnant SD rats were randomly divided into three groups. SD rats in the control group (CON group) were intraperitoneally injected with phosphate buffered saline (PBS) on the 17^th^ and 18^th^ embryonic days (E17 and E18), and corn oil on the 19^th^ embryonic day (E19). In contrast, SD rats in the model group (PVL group) were intraperitoneally injected with 500 µg/kg LPS (*Escherichia coli*, Serotype 055: B5, Sigma) on E17 and E18, and corn oil on E19. SD rats in the selective A_2B_AR antagonist group (PVL-PSB group) were intraperitoneally injected with LPS on E17 and E18, and 10 µg/kg PSB0788 (Tocris Bioscience) on E19. Seven-day-old rats (P7) were subjected to the following treatments, taking no account of their gender.

### 2.3 Immunohistochemistry

Seven-day-old rats (P7) were anesthetized by intraperitoneal injection of pentobarbital sodium (50 mg/kg) and fixed *in situ* by intracardiac perfusion with 4% paraformaldehyde. The whole brain was removed and subsequently embedded in paraffin for tissue sectioning. The 5 µm paraffin sections were dewaxed and brough into water through a graded ethanol series. Antigen retrieval was performed in 0.01 M citrate buffer (pH 6.0) in a microwave oven. The sections were blocked with goat serum and incubated for 12 h at 4°C with primary antibody (Rat mAb to MBP, 1:200 dilution, Abcam AB7349; Rb pAb to NG2, 1:100 dilution, Abcam ab129051). The sections were then washed in PBS, incubated at room temperature for 1 h with the secondary antibody (HRP Goat Anti-Rat IgG, 1:400 Dilution, Abbkine A21040; HRP Goat Anti-Rabbit IgG 1:400 Dilution, Abbkine A21020), and washed again. After diaminobenzidine (DAB) and hematoxylin staining, the nuclei were observed under a light microscope.

### 2.4 Immunofluorescence staining

Sections were prepared as for immunofluorescence, and incubated with primary antibody at 4°C for 12 h (Mouse mAb CC-1 1:100 dilution, Calbiochem OP80-100ug; Rb mAb to Olig2, 1:100 dilution, Abcam AB109186), and then incubated at room temperature for 1 h in the dark with the second antibody (Dylight 594 Rabbit IgG, 1:300 dilution, Abbkine A23420; Dylight 488 Mouse IgG 1:300 dilution Abbkine A23210). Cell nuclei were stained with 4’, 6-diamidino-2-phenylindole (DAPI). Fluorescence values were measured by a fluorescence microscope(Olympus BX53, Olympus, Japan).

### 2.5 Western blot

The offspring at P7 of the injected rats were anesthetized by intraperitoneal injection of sodium pentobarbital, decapitated, and the cerebral white matter rapidly separated. Total protein was extracted with protein lysis buffer (Keygentec), and protein concentration was measured. Samples with equal amounts of protein (30 µg) were loaded on sodium dodecyl sulfate polyacrylamide gels for electrophoresis (Bio-Rad, CA, USA) and transferred onto 0.45 µm PVDF membranes. The membranes were incubated at 4°C overnight with different primary antibodies (Rat mAb to MBP, 1:1000 dilution, Abcam ab7349; Rb pAb to NG2, 1:1000 dilution, Abcam ab129051; β-Tubulin mouse antibody, 1:5000 dilution, Multi Sciences ab009-100; MS mAb to β-Actin, 1:5000 dilution, Origene TA-09), and subsequently labeled with appropriate secondary antibodies (HRP Goat anti-rabbit IgG, 1: 5000 dilution, Abbkine A21020; HRP Goat anti-rat IgG, 1: 5000 dilution, Abbkine A21020; HRP Goat anti-mouse IgG, 1: 5000 dilution, Abbkine A21010) for 1 hour at room temperature. The protein signals were visualized using an enhanced chemiluminescence (ECL) kit (Millipore, USA) in a ECL imaging system (Syngene G: BOX, UK). Quantification of protein bands was performed using ImageJ software.

### 2.6 ELISA

At P7, offspring rats were anesthetized by intraperitoneal injection of pentobarbital sodium, decapitated, and the cerebral white matter rapidly separated. The concentrations of IL-1 β, IL-6 and TNF-α in the cerebral white matter of rats was determined by the corresponding ELISA kit (Jiangsu Jingmei Biological Technology Co., Ltd.,China) according to the manufacturer’s instructions. After processed, the samples were added into the plate, and the absorbance at 450 nm was repeatedly read using a spectrophotometer (SpectraMax, Thermo, USA).

### 2.7 Transmission electron microscopy (TEM)

The offspring rats were anesthetized by intraperitoneal injection of pentobarbital sodium (50 mg/kg) at P7 and perfused with cold 4.0% glutaraldehyde in PBS (pH 7.4) through the heart. A sagittal incision was made on the brain. The samples are dehydrated through sequential passes through 50%, 70%, 80%, 90%, 95%, 100%, and 100% alcohols for about 30 minutes each. The samples were then incubated in a mixed solution of acetone and embedding medium (1:1 ratio) overnight, and polymerized at 60°C for 48 h. The final block was cut into ultrathin sections (60–80 nm thickness). The morphology of oligodendrocytes was observed under TEM.

### 2.8 Statistical analysis

All statistical analysis was performed using GraphPad Prism Version 8.0 (GraphPad Software Prism, La Jolla, CA, USA) and SPSS Version 22.0 (IBM SPSS Version 22, Chicago, IL). All the data were reported as mean ± SD. The continuous data in groups was compared by student’s t-test. The categorical data was analyzed by χ2 test. P < 0.05 was considered statistically significant.

## 3 Results

In this study, it was hypothesized that PSB0788 ameliorates white matter injury via promoting the expression of IL‐10.The aim of the study was to discover new targets for the treatment of PVL. The goal of this study was to prove that PSB0788 could improve the myelination disturbances caused by maternal inflammation‐induced PVL.

### 3.1 Intrauterine infection in pregnant rats caused PVL in offspring rats

Based on the method by Tuzun et al., intraperitoneal injection of LPS was administered consecutively on E17 and E18 in pregnant rats to establish the PVL model in their offspring [28]. Changes in oligodendrocytes and myelin sheath were observed in offspring rats at P7 (Figure 1(a)). Figure 1(b) shows the markers at different developmental stages from OPCs to myelinating oligodendrocytes. OPCs were characterized by the expression of chondroitin-sulfate proteoglycan (NG2 Proteoglycan, NG2) in the cytoplasm [29]; adenomatous polyposis coli (APC, CC-1) was used as a marker of mature oligodendrocytes [30]; the differentiated myelinating oligodendrocytes were characterized by MBP [31,32]. The samples of offspring rats at P7 were collected from the shoulder of the corpus callosum around the ventricle (Figure 1(c)).

**Figure 1.** (a) After the *in vivo* PVL model was established, changes in oligodendrocytes were observed in offspring rats at P7. (b) The black line is the coronal section, and the box represents the detection area.

Placental inflammation was observed by H&E staining. Lymphocytes and neutrophils infiltrated through the vascular wall of the placenta in the PVL group, while no inflammatory cells were observed in the vascular wall of the placenta in the CON group (Figure 2(a)). The levels of IL-1 β, IL-6, and TNF‐α in the brain tissue of the offspring rats at P7 in the PVL group were found to be significantly increased by ELISA (Figure 2(b)). PVL can cause myelination disorders in newborns [33]. We verified the level of MBP in offspring rats at P7 through immunohistochemistry (Figure 3(a)) and western blot (Figure 3(b)), and the results showed that the expression of MBP in the PVL group was significantly lower than that in the CON group.

**Figure 2.** The offspring rats in the PVL group showed signs of inflammation. (a) H&E staining showed the infiltration of inflammatory cells in the vascular wall of a placenta from the PVL group.*Scale bar*.50 μm. (b) The results of ELISA showed that the expression of inflammatory cytokines IL-1 β, IL-6 and TNF-α was increased in the PVL group. Data were expressed as mean ±SD (n = 5). ^#^*P < *0.05 for student’s t-test.

**Figure 3.** PVL lead to low expression of MBP. (a) Immunohistochemical results showed that the number of MBP positive cells in the shoulder area of the corpus callosum in the PVL group was significantly reduced compared to the CON group.*Scale bar*.100 μm. (b) The level of MBP protein in the cerebral white matter of offspring rats in the PVL group was significantly decreased. Data were expressed as mean ±SD (n = 5). ^#^*P < *0.05 for student’s t-test.

### 3.2 Maternal inflammation‐induced PVL reduced the number of OPCs and mature oligodendrocytes in offspring rats

We observed a decreased myelination rate in the PVL group. The results of immunohistochemistry (Figure 4(a)) and western blot (Figure 4(b)) showed that the expression level of NG2 in the PVL group was significantly lower than that in the CON group, indicating a significant decrease in the number of OPCs in offspring rats. We identified the number of mature oligodendrocytes through double-labeling by immunofluorescence (CC-1/Olig2), and the results showed that their number in the PVL group was significantly lower than that in the CON group (Figure 4(c)). In TEM, oligodendrocytes were found to have in oval nuclei in the CON group, with complete and visible nuclear membrane, and evenly distributed chromatin; while the nuclei of oligodendrocytes in the PVL group were irregular in morphology, with discontinuous nuclear membrane, and decreased chromatin (Figure 4(b)).

**Figure 4.** PVL could affect the development and differentiation of OPCs in offspring rats. (a) Immunohistochemistry showed that the number of NG2 positive cells in the shoulder of the corpus callosum in the PVL group were significantly fewer than in the CON group.*Scale bar*.20 μm. (b) The results of western blot showed that the level of NG2 protein in the cerebral white matter of offspring rats in the PVL group was significantly decreased. (c) The results of immunofluorescence staining showed that the number of CC-1/Olig2 positive cells in the shoulder of the corpus callosum decreased significantly in the PVL group.*Scale bar*.100 μm. (d) Transmission electron microscopy revealed damaged oligodendrocytes cells in the PVL group.*Scale bar*.2 μm. Data were expressed as mean ±SD (n = 5). ^#^*P < *0.05 for student’s t-test.

### 3.3 Selective A_2B_AR antagonist PSB0788 promoted myelin-associated glycoprotein expression in offspring rats

Figure 5(a) shows that pregnant rats in PVL model were further injected at E19 with PSB0788, a selective A_2B_AR antagonist. After PSB0788 treatment during pregnancy, the expression of MBP in was higher than in the PVL-CON group, through immunohistochemistry (Figure 5(b)) and western blot (Figure 5(c)).

**Figure 5.** PSB0788 treatment increased MBP expression. (a) Intraperitoneal injection of PSB0788 at E19 was performed to observe changes in oligodendrocytes at all stages in brains of offspring rats at P7. (b) Immunohistochemical results showed that the number of MBP positive cells in the shoulder of the corpus callosum in the PVL-PSB group was significantly increased compared to the PVL-CON group.*Scale bar*.100 μm. (c) The results of western blot showed that the level of MBP protein in the cerebral white matter of offspring rats in the PVL-PSB group was increased significantly. Data were expressed as mean ±SD (n = 5). ^#^*P < *0.05 for student’s t-test.

### 3.4 Effect of selective A_2B_AR antagonist PSB0788 on the differentiation of OPCs in demyelinated in offspring rats

The results of immunohistochemistry (Figure 6(a)) and western blot (Figure 6(b)) showed that the expression level of NG2 in the PVL-PSB group was increased compared to the PVL-CON group. This is consistent with immunofluorescence staining showing that the number of CC-1/Olig2 positive cells in the PVL-PSB group was higher than in the PVL-CON group (Figure 6(c)). TEM showed that the nuclei of oligodendrocytes in the PVL-PSB group were oval, with complete membrane and increased organelles (Figure 6(d)).

**Figure 6.** PSB0788 treatment of PVL promoted the development and differentiation of OPCs. (a) The number of NG2 positive cells in the shoulder of the corpus callosum in the PVL-PSB group was higher than in the PVL-CON group. *Scale bar*.20 μm.(b) NG2 protein level increased in the cerebral white matter of offspring rats in the PVL-PSB group. (c) The number of CC-1/Olig2 positive cells in the shoulder of the corpus callosum increased in the PVL-PSB group. *Scale bar*.100 μm.(d) Oligodendrocytes in the PVL-PSB group tended to be normal.*Scale bar*.2 μm. Data were expressed as mean ±SD (n = 5). ^#^*P < *0.05 for student’s t-test.

### 3.5 Selective A_2B_AR antagonist PSB0788 promoted the expression of IL‐10

ELISA showed that cytokines IL-1 β, IL-6, and TNF‐α in the PVL-PSB group were not significantly different from those in the PVL-CON group, but IL-10 was significantly increased in the PVL-PSB group (Figure 7(a)).

**Figure 7.** PSB0788 treatment activated anti-inflammatory microglia. (a) The level of inflammatory cytokines IL-1 β, IL-6 and TNF-α were not significantly different in the PVL-PSB group from those in the PVL-CON group, while IL-10 was significantly increased in the PVL-PSB group. ^#^*P < *0.05 for student’s t-test.

## 4. Discussion

Infection during pregnancy has been recognized as an important cause of PVL [34]. Inflammation-induced PVL causes an upregulation of pro-inflammatory cytokines. Inflammation-induced brain injury spread by consistent inflammation, impacted on differentiation of oligodendrocyte subpopulations, axonal growth and myelination. Myelination disturbances in cerebral white matter are related to aberrant regeneration and repair responses to the acute death of cells in oligodendrocyte subpopulations, especially OPCs [35,36]. On the other hand, Kim et al. found that intracerebroventricularly transplantation with OPCs in PVL rats could promote myelination or myelin regeneration, thus restoring neurobehavioral functions by preventing axonal demyelination to a certain extent [37]. Based on the results of previous studies, intraperitoneal injection of LPS was administered consecutively at E17 and E18 in pregnant rats to induce intrauterine infection and establish the PVL model in their offspring [38–40]. In line with this, our experiment revealed high expressions of IL-1β, IL-6 and TNF-α in the cerebral white matter of offspring rats, which is also a common feature of the inflammation-induced PVL model [9]. As maternal inflammation disrupted white matter development in the growing brain and reduced the number of OPCs, the offspring rats lead to white matter‐related injuries and impaired neurological function [41,42], which was consistent with the results of our study. Pro-inflammatory cytokines such as IL-1β and TNF-α influenced on the myelin sheath by killing OPCs and inhibited the maturation of oligodendrocytes [43–45].In the present study, PVL model, disturbed the myelination process indicated by a decrease in the expression of NG2, CC-1 and MBP.

Prenatal treatment avoids disease to prompt serious and incurable injuries in the fetus.This novel approach has become a new prospect in congenital disorders. PSB0788 is a fat-soluble drug [26] that can be easily absorbed by the embryo across the placental barrier. Therefore, intraperitoneal injection of PSB0788 was administered to pregnant rats to treat potential PVL in offspring rats. The results showed that the expressions of NG2, CC-1, and MBP in offspring rats were significantly increased after prenatal treatment of PSB0788, indicating that PSB0788 could increase the level of OPCs and mature oligodendrocytes, thus alleviating the symptoms of demyelination caused by infection, and improving the adverse effects of prenatal inflammation on offspring cerebral white matter.

Particularly, preterm infants are susceptible to inflammatory disorders because of the sensitivity to program that constantly affects development. Modulating the inflammatory cytokines secretion is a contributing piece of therapeutic strategies.Merighi et al showed that inhibiting A_2B_AR lessens the IL‐6 production in spinal cord injury [46].In the present study, we utilized PSB0788, which is a selective A_2B_AR antagonist, for prenatal treatment of PVL. Our data showed that maternal inflammation caused an elevation in proinflammatory cytokines, whereas intraperitoneal injection of PSB0788 into the pregnant mice increased the expression of anti-inflammatory cytokines in protein levels. Actually, Li et al. found that IL-10 elevated numbers of OPCs and oligodendrocytes through mechanisms that involved both immunomodulation and induction of neurotrophic factors in the demyelination model [47]. In this study, we believe that psb0788 can improve the remyelination by increasing the expression of IL-10, and the remyelination can be indicated by the increase of MBP protein.

Therefore, we believe that PSB0788 could improve the myelination disturbances caused by PVL, acting to treat neonatal neurologic diseases. This study is still have some limitations. Future studies of immune function and mechanism will be important for showing potentially therapeutic targets to prevent injury secondary to PVL and revealing the consequences of immune changes to injuries through the lifespan.

## 5. Conclusion

The findings of our study provide a promising strategy for the treatment of maternal inflammation‐induced PVL. In this model, the selective A_2B_AR antagonist PSB0788 played an important role in promoting the development and differentiation of OPCs. In subsequent studies, we will focus on the mechanism of action of PSB0788 in maternal inflammation‐induced PVL.
